This article has been retracted.

# Extremely Active Nano-formulation of Resveratrol (XAR™) attenuates and reverses chemotherapy-induced damage in mice ovaries and testes

**DOI:** 10.1186/s13048-022-01043-8

**Published:** 2022-10-21

**Authors:** Sagar Chhabria, Vaishnavi Takle, Nripen Sharma, Prashant Kharkar, Kshama Pansare, Anish Tripathi, Ashish Tripathi, Deepa Bhartiya

**Affiliations:** 1 Epigeneres Biotech Pvt. Ltd., Sun Mill Compound, Ikon House, B-Block, Senapati Bapat Marg, Lower Parel, Mumbai, Maharashtra 400013 India; 2 Department of Pharmaceutical Sciences and Technology, Institute of Chemical Technology, Matunga, Mumbai, 400 019 India; 3 Shobhaben Pratapbhai Patel School of Pharmacy & Technology Management, SVKM’s NMIMS, Vile Parle (West), Mumbai, 400 056 India

**Keywords:** Ovary, Testis, Stem cells, Very small embryonic-like stem cells (VSELs), Chemotherapy, Infertility, Premature ovarian failure, Spermatogenesis

## Abstract

**Background:**

Fertility preservation and restoration in cancer patients/survivors is the need of present times when increased numbers of patients get cured of cancer but face infertility as a serious side effect. Resveratrol has beneficial effects on chemoablated ovaries and testes in mice but has failed to enter the clinics because of extremely poor bioavailability. The present study was undertaken to evaluate the protective and curative effects of Extremely active Resveratrol (XAR™)- a nano-formulation of resveratrol with significantly improved bioavailability- on mouse ovary and testis after chemotherapy. Effects of XAR™ and FSH were compared on stimulation of follicle growth in adult mice ovaries. XAR™ (25 mg/kg) was administered for two days prior to chemotherapy to study the protective effects on the mouse gonads. XAR™ was also administered for 14 days post chemoablation to study the regenerative effects. Besides effect on numbers of primordial and growing follicles and spermatogenesis, the effect of XAR™ was also evaluated on the transcripts specific for ovarian/testicular stem/progenitor/germ cells, their proliferation, differentiation, meiosis, and the antioxidant indices.

**Results:**

Similar to FSH, XAR™ increased the numbers of primordial follicles (PF) as well as growing follicles. It protected the gonads from the adverse effects of chemotherapy and showed the ability to regenerate non-functional, chemoablated gonads. Besides stimulating follicle growth in adult ovaries similar to FSH, XAR™ also protected the testes from the adverse effects of chemotherapy and improved spermatogenesis. This was accompanied by improved anti-oxidant indices.

**Conclusions:**

The results of the present study potentiate the use of XAR™ in pilot clinical studies to protect gonadal function during oncotherapy and also regenerate non-functional gonads in cancer survivors by improving antioxidant indices and stem cell-based tissue regeneration.

**Supplementary Information:**

The online version contains supplementary material available at 10.1186/s13048-022-01043-8.

## Background

Cancer is the second leading cause of death globally and is responsible for an estimated 10 million deaths in 2020 [1]. While the incidence of cancer continues to increase, fortunately, cancer survivorship is also on the rise due to improved detection and treatment protocols [2]. Chemotherapeutic drugs are potent and efficient in fighting cancer; they also exert debilitating side effects on various organs including the gonads [3, 4]. Chemotherapy-induced compromised infertility in young male and female survivors is now acknowledged as one of the most destructive long-term adverse effects [5]. Chemotherapy is known to cause irreversible ovarian and testicular damage that puts females and males at the risk of premature ovarian failure and azoospermia respectively [3, 6]. The risk of chemotherapy-induced infertility has been reported to be in around 80% of cases [7]. Therefore, it is becoming increasingly important to address concerns about the long-term effects of chemotherapy and explore potential fertility reversion options for cancer patients.

Bhartiya [8] reviewed published literature on the effects of oncotherapy on endogenous, tissue-resident gonadal stem cells wherein pluripotent very small embryonic-like stem cells (VSELs) survive oncotherapy, almost double in numbers after chemotherapy in both mouse ovaries and testes and can be manipulated to regenerate the non-functional gonads. The stem cells niche gets compromised by oncotherapy and transplanting autologous bone marrow derived mesenchymal cells helps to restore gonadal function and this approach has also resulted in the birth of fertile pups. The VSELs are pluripotent stem cells that exist in multiple adult tissues, give rise to tissue specific stem cells ‘progenitors’ including spermatogonial stem cells (SSCs) in testis and ovarian stem cells (OSCs) in ovaries and were recently reviewed [9–11]**.** VSELs undergo rare asymmetrical cell divisions to self-renew and give rise to slightly bigger progenitors that in turn undergo symmetrical cell divisions and clonal expansion prior to initiating differentiation [12].

Resveratrol (3,5,4′-trihydroxy-trans-stilbene), a natural anti-oxidant and phytoestrogen molecule present in grapes, mulberries, groundnuts and red wine etc. is known to delay ageing by acting on multiple organs, by improving DNA repair and protein function, cellular detoxification and energy production [13]. Several reports have discussed the preventive effects of resveratrol against neuro-degeneration, ovarian dysfunction, infertility, muscular dystrophy, diabetes, cancer and other ageing ailments in animal models [14–17]. Wu et al. reported that intraperitoneal administration of resveratrol promoted spermatogonial stem cells (SSC) proliferation in testis and furthermore led to the cessation of SSC loss in azoospermia mice model [18]. Yulug et al. [19] reported the protective effect of intraperitoneally administered resveratrol against methotrexate induced testis damage in rats. Kong et al. [20] discussed that resveratrol injection could effectively regulate ovarian development. Bioavailability of resveratrol remains a key challenge for it to enter the market. More than 14,000 sirtuin activators have now been identified [21] with the hope to find a molecule with enhanced bioavailability.

We have earlier reported a direct action of XAR™ on stem cells in human blood [22]. The tissue-resident VSELs express pluripotent markers along with ERα, ERβ and FSHR in multiple tissues [23, 24] and thus it was of interest to study if XAR**™** could exert similar effects like FSH on the ovaries. In the present study, the effects of XAR™ and FSH were compared on numbers of primordial and growing follicles in adult mouse ovary and correlated with circulatory levels of Anti Mullerian Hormone (AMH). In addition we studied, the protective and curative effects of XAR™, to restore gametogenesis in chemoablated testes and ovaries along with improvement of antioxidant indices in circulation.

## Study design and methods

The study protocol of the current investigation was approved by the Institutional Animal Ethics Committee of SVKM’s NMIMS University, Mumbai, India (IAEC/P-16/2017). 6–8 weeks old female and male mice were housed at the central animal facility at SVKM’s NMIMS University, Mumbai, India under standard conditions and with free access to food and water. They were housed in a temperature and humidity-controlled room on a 12h light and 12h dark cycle. The animals were divided into three treatment groups viz. Group A, B & C (Fig. 1).

**Fig. 1:** Schematic representation of the experimental design and group composition. The study comprises of 3 groups; evaluating the effects of FSH and XAR™ formulation on mouse ovaries in Group A and the curative preventive effects of XAR™ treatment after chemotherapy in females – Group B and males – Group C. Group A comprises of 5 sub-groups; control, mice treated with only FSH for 2 and 4 days, and with only XAR™ formulation for 2 and 4 days respectively. The mice were sacrificed on Day 7. Group B for female mice chemoablation studies comprises of 6 sub-groups; control, mice treated with only XAR™ formulation, curative control – Busulfan (Bu) – Cyclophosphamide (Cy) treatment, curative treatment – post 30 days of Bu-Cy treatment, the XAR™ treatment was continued for 2 weeks, preventive control—Bu-Cy treatment and preventive treatment—Bu-Cy- XAR™ treatment, wherein XAR treatment was initiated 2 days prior to Bu-Cy and continued until Day 30. Group C for male mice chemoablation studies comprises of 6 sub-groups; control, mice treated with only XAR™ formulation, curative control – only Bu treatment, curative treatment – post 30 days of Bu treatment, the XAR™ treatment was continued for 2 weeks, preventive control—Bu treatment and preventive treatment—Bu-Cy- XAR™ treatment, wherein XAR treatment was initiated 2 days prior to Bu and continued until Day 30. In Group B and C, the mice were sacrificed as per the defined end-point on Day 30 or Day 45

Epigeneres Biotech Private Limited, Mumbai, India has a patented formulation, a bio-stabilized nano-formulation XAR™ using principles of nanotechnology and bio-mimicry to enhance the bioavailability of resveratrol, for human consumption and will be made available to any group upon request. Dose for administration to mice in the present study was calculated based on earlier report discussing dose equivalence [25]. Commercially available recombinant human FSH (Gonal F) was used to treat the mice using similar dose as reported earlier [26].

### Effects of FSH and XAR™ treatment on mouse ovaries

Group A consisted of 60 eight weeks old female mice. They were randomly divided into five groups, each group consisting of 12 animals. Control group was not subjected to any treatment. FSH D2 group was injected 5U of FSH per mouse intraperitoneally for two days. FSH D7 group was injected with 5U of FSH for four days and the animals were sacrificed after three days. XAR™ D2 group received XAR™ (25 mg/kg) via oral gavage for two days. XAR™ D7 group was administered XAR™ (25 mg/kg) orally for four days and the animals were sacrificed after three days.

### Curative and preventive effects of XAR™ after chemotherapy in female mice

Group B consisted of 72 eight weeks old female mice. They were randomly divided into six groups, each group consisting of 12 animals. All the mice, except the control group and XAR™ group, were treated with Busulfan (Bu) 10 mg/kg daily for four days and 100 mg/kg cyclophosphamide (Cy) for the first two days through the intraperitoneal route. Busulfan (Sigma-Aldrich, Missouri) was dissolved in dimethyl sulfoxide (Sigma-Aldrich), diluted with equal volume of sterile water and injected via the intraperitoneal route. Cyclophosphamide (Baxter, India) was dissolved in sterile injection grade water and injected via the intraperitoneal route after 2 h of busulfan injection. This treatment regimen has earlier been reported to induce chemoablation of mouse ovaries [26]. The control group was not subjected to any treatment. XAR™ group received XAR™ (25 mg/kg) orally for 45 days. The Curative Bu-Cy control group was treated with Bu-Cy and later sacrificed on D45. Curative Bu-Cy-XAR™ group was administered XAR™ (25 mg/kg) orally after 30 days of Bu-Cy for two weeks and then mice were sacrificed on D45. To study the protective/preventive effect of XAR™, the treatment with XAR™ was initiated two days prior to Bu-Cy treatment and the preventive control group received only Bu-Cy (chemotherapy) and no XAR™. Both the groups were sacrificed on D30.

### Curative and preventive effects of XAR™ after chemotherapy in male mice

Group C consisted of 72 eight weeks old male mice. They were randomly divided into six groups, each group consisting of 12 animals. All the mice, except the control group and XAR™ group, were treated with Busulfan (Bu) 25 mg/kg daily for four days through the intraperitoneal route. The control group was not subjected to any treatment. XAR™ group received XAR™ (25 mg/kg) orally for 45 days. The curative control group was treated with Bu and later sacrificed on D45. Curative Bu-XAR™ group was administered XAR™ (25 mg/kg) orally after 30 days post Bu treatment for two weeks and then sacrificed on D45. To study the protective effect of XAR™, control group received Bu and sacrificed on D30 whereas the Bu-XAR™ group was administered XAR™ two days before Bu and mice were sacrificed on D30 after Bu treatment.

#### Processing of tissues for various studies

##### Histology

Ovaries and testes were collected from various treatment groups, weighed and fixed in neutral buffered formalin for histological studies. Standard methods were used to make paraffin blocks and 5 μm sections were prepared for various studies.

##### Follicle count

Ovaries were fixed in Bouin’s fixative, then embedded in paraffin in an automated tissue processor. Whole ovaries were serially cut from cortex into 5 μm sections. Every fifth section was subjected to hematoxylin and eosin staining. Counting was performed while being double-blinded to treatment conditions or groups. The Panoramic 250 Flash Slide Scanner system (3D Histech, Budapest, Hungary) was used to capture digital whole-slide high-resolution images with an X40 Plan-Apochromat objective and an X1.6 camera adapter magnification. The follicle stage was classified according to accepted definitions [27].

##### Sperm count

To determine the sperm count in various groups, sperm were collected from cauda epididymis and transferred to pre-warmed saline (37 °C). A longitudinal incision was made using a fine needle and scalpel blade to release sperm. The epididymis was incubated for 10 min at 37 °C to allow the sperm to swim out of the epididymal tubules. The total number of sperm and motile sperms were determined using hemocytometer, the sperm motility was converted into a percentage.

##### Hormone analysis

The blood samples collected by retro-orbital puncture was allowed to clot at room temperature and centrifuged to harvest serum. Serum biochemical parameters such as serum follicle stimulating hormone (FSH), luteinizing hormone (LH), progesterone (P), estradiol (E_2_), AMH and testosterone (T) were analysed spectrophotometrically (Shimadzu, Kyoto, Japan) using commercially available ELISA kits for FSH (Novus Biologicals, Littleton, USA KA2330), LH (Novus Biologicals, Littleton, USA KA2332), P (Cayman Chemicals, Ann Arbor, MI, USA 582,601), E_2_ (Cayman Chemicals, Ann Arbor, MI, USA 582,251), AMH (Abbkine, Hubei, China KTE71557) and T (Abcam 108,666, USA).

##### RNA isolation and cDNA synthesis

Total RNA was extracted from the tissues placed in Trizol (Invitrogen) and was treated with DNase I (Amersham Biosciences; Piscataway, NJ) to remove any genomic DNA contamination. First-strand cDNA was synthesized using the Revert Aid First strand cDNA synthesis kit (Thermo Fisher Scientific, UK) according to the manufacturer’s instructions. Briefly, 1 μg of total RNA was incubated with 5X Reaction Buffer and reverse transcriptase mix. The reaction was carried out in Applied Biosystems GeneAmp® thermal cycler 9700 (Applied Biosystems, USA) as per the manufacturer’s instructions.

##### qRT-PCR studies

The expression levels of various gene transcripts specific for stem cells (*Oct-4A, Sox-2, Nanog, Sca1*), progenitors (*TOct-4*), primordial germ cells (*Stella, Fragilis*), germ cells (*MVH, Gfra, Dazl, c-kit, cyclin B1, Nobox Hoxa10*), proliferation (*PCNA*), pre-meiotic (*Stra8*), meiotic (*Scp3, Dmc1, Stra8, Prohibitin*), post-meiotic (*Protamine*), FSH receptors (*Fshr1, Fshr3*) and antioxidant indices (*Sirt1, Sirt6, Nampt, p53*) were estimated by real-time PCR system-ABI 7500 (Applied Bio-systems, USA) using gene specific primers and Thermo Scientific Maxima SYBR Green/ROX qPCR Master Mix kit (Thermo scientific, UK). The 18 s rRNA gene was used as the housekeeping gene. The primers used in the study and reasons to study them are mentioned in Supplementary Table 1. The amplification conditions were: initial denaturation at 94 °C for 3 min followed by 40 cycles comprising of denaturation at 94 °C for 10 s, primer annealing for 20 s, and extension at 72 °C for 30 s followed by melt curve analysis to determine homogeneity of the PCR amplicons. C_t_ values generated in each experiment using the 7500 Manager software (Applied Bio-systems, UK) were used to calculate the mRNA expression levels. The fold change was calculated using ΔΔC_t_ method. In all qRT-PCR experiments, the value of average fold change has been calculated with respect to chemoablated control group.

##### Measurement of antioxidant indices

The antioxidant indices such as Superoxide Dismutase (SOD) (ab65354), Glutathione Peroxidase (GSH-Px) (ab102530), Malondialdehyde (MDA) (ab118970) were analysed in the tissues using commercial biochemical kits as per the manufacturers protocol (Abcam, MA, USA).

##### Statistical analysis

The mean and standard deviation were calculated for all the groups. All the data were analysed for statistical significance using GraphPad Prism software ver. 8.4.2 (San Diego, CA, USA). Differences between groups were considered statistically significant when *p* < 0.05.

## Results

### Effects of FSH and XAR™ treatment on adult mice ovaries

As shown in Table 1A, the number of both primordial and growing follicles were increased after treatment with FSH as well as with XAR™ in Group A. It is intriguing to note as compared to FSH D7 the effect of XAR™ was more on primordial follicles on Day 7 rather than on the growing and antral follicles. Moreover, XAR**™** treatment on D7 led to statistically significant increase (*p* < 0.01) in AMH levels when compared to untreated control whereas FSH treatment led to no significant effect in the AMH levels compared to untreated control. Atretic follicles were not enumerated since focus of present study was on growing follicles due to FSH and XAR**™** treatment.

**Table 1:** Effect of XAR^TM^ treatment on chemoablated ovary and testis. **A**. Effect of FSH and XAR™ treatment on adult mouse ovary. The FSH treatment led to increased levels of primordial, growing and antral follicles in both Day 2 and Day 7 group, while the XAR™ treatment led to a significant increase in the growing and antral follicles in Day 2 group, and primordial, growing and antral follicles in Day 7 group. An increase in AMH levels was also observed in XAR™ treated Day 7 group. **B**. Curative and preventive effects of XAR™ on circulatory levels of hormones in adult female mice. XAR™ treatment led to increased AMH, progesterone, estrogen levels and decreased FSH and LH levels in chemoblated mice. **C**. Curative and preventive effect of XAR™ on circulatory levels of hormones in adult male mice. The decreased levels of testosterone, sperm count, sperm viability and sperm motility in chemoblated mice, were restored to normal levels on XAR™ treatment, in both preventive and curative group. Two-way ANOVA was used for statistical analysis, ^####^*p* < 0.0001, ^###^*p* < 0.001, ^##^*p* < 0.01, ^#^*p* < 0.05. The hash sign (^#^) indicates statistically significant difference between untreated control and the indicated groups, while the asterisk sign (*) indicates statistical significance within the treatments. “ns” indicates statistically non-significant differences

**A: Comparing effect of FSH and XAR™ treatment on adult mouse ovary**						
**Groups**		**Primordial**	**Growing**	**Antral**	**AMH values** **(ng/ml)**	
Untreated Control		144 ± 11	94 ± 8	48 ± 5	16.10 ± 1.5	
FSH treated Day 2		192 ± 20^##^	159 ± 13^###^	131 ± 16^####^	-	
FSH treated Day 7		198 ± 21^##^	181 ± 19^####^	135 ± 14^####^	20.84 ± 2.1^ ns^	
XAR™ treated Day 2		148 ± 15^ ns, *^	119 ± 12^ ns, *^	81 ± 9^#, **^	-	
XAR™ treated Day 7		254 ± 24^####, ***^	152 ± 18^###^	83 ± 10^#, **^	24.35 ± 2.5^##^	
**B. Curative & preventive effects of XAR™ on circulatory hormones in female mice**						
**Hormones**	**Untreated** **Control**	**XAR™ treatment**	**Bu-Cy** **Curative Control**	**Bu-Cy XAR™** **Curative treatment**	**Bu-Cy** **Preventive Control**	**Bu-Cy XAR™** **Preventive treatment**
FSH (ng/ml)	0.55 ± 0.04	0.84 ± 0.09^ ns^	1.98 ± 0.21^####^	0.86 ± 0.08^ ns, ****^	1.45 ± 0.17^####^	0.63 ± 0.07^ ns, ****^
LH (ng/ml)	2.92 ± 0.24	3.18 ± 0.36^ ns^	5.42 ± 0.58^####^	3.99 ± 0.44^ ns, *^	4.74 ± 0.50^##^	3.36 ± 0.39^ ns, *^
P (pg/ml)	41.24 ± 3.98	44.39 ± 5.01^ ns^	11.29 ± 1.55^####^	34.53 ± 5.98^ ns, ***^	17.34 ± 3.01^###^	36.46 ± 4.91^ ns, **^
E_2_ (pg/ml)	261.34 ± 31.95	274.46 ± 34.15^ ns^	139.45 ± 15.49^##^	211.54 ± 26.08^ ns, *^	163.35 ± 18.84^##^	256.28 ± 29.98^ ns, *^
AMH (ng/ml)	16.10 ± 2.09	31.39 ± 4.58^####^	3.59 ± 0.42^###^	15.24 ± 1.17^ ns, ***^	6.49 ± 0.59^##^	18.93 ± 1.96^ ns, ***^
**C. Curative & preventive effects of XAR™ on circulatory hormones in male mice**						
**Hormones**	**Untreated Control**	**XAR™** **treatment**	**Bu Curative** **Control**	**Bu- XAR™ Curative treatment**	**Bu Preventive Control**	**Bu- XAR™ Preventive Treatment**
Testosterone (ng/ml)	4.31 ± 0.41	4.56 ± 0.46^ ns^	1.56 ± 0.2^####^	4.09 ± 0.43^ ns, ****^	2.06 ± 0.25^###^	4.16 ± 0.58^ ns, ***^
Sperm Count (10^6^/ ml)	22.93 ± 3.2	24.56 ± 2.9^ ns^	1.39 ± 0.19^####^	19.87 ± 2.1^ ns, ***^	1.99 ± 0.22^####^	20.49 ± 2.9^ ns, ***^
Sperm Motility (%)	86.29 ± 9.3	89.93 ± 9.1^ ns^	16.83 ± 1.8^####^	76.39 ± 8.3^ ns, ****^	21.27 ± 2.5^####^	74.87 ± 6.9^ ns, ****^
Sperm Viability (%)	76.32 ± 8.3	78.38 ± 8.2^ ns^	13.29 ± 1.4^####^	69.39 ± 7.5^ ns, ****^	10.39 ± 1.2^####^	72.39 ± 8.8^ ns, ****^

### Effect of treatment on the weight of gonads

Post 45 days of XAR™ treatment, the weight of the gonads was maintained in the mice. Chemoablation (with Cy + Bu in female and Bu in male mice) resulted in more than two-fold reduction (*p* < 0.05) in ovary and testis weight which was evidently recovered (*p* < 0.05) by XAR™ treatment for 15 days. Interestingly, loss of weight of both ovary and testis was prevented (*p* < 0.05) after chemotherapy, by prior treatment with XAR™ for 30 days (Fig. 2).

**Fig. 2:** Curative and protective effects of XAR™ treatment on adult ovaries and testis. The weight of (**A**) adult ovaries and (**B**) testis decreased in both curative and preventive control groups treated with Bu-Cy treatment in female mice and Bu treatment in male mice. On treatment with XAR™ formulation, both the adult ovaries and testis regained significant weight in Bu-Cy and Bu treated mice, suggesting the curative and preventive effect of XAR™. Compared to control, the mice treated only with XAR™ formulation, showed no difference in weight. Two-way ANOVA was used for statistical analysis, ****p < 0.0001, ***p < 0.001, **p < 0.01, *p < 0.05

## Effect of XAR™ on circulatory levels of hormones in chemoablated mice

Table 1B and C show circulatory levels of pituitary and steroid hormone levels in both female (Table 1B) and male (Table 1C) mice along with sperm parameters. As evident in Table 1B levels of AMH were statistically raised (*p* < 0.0001) after XAR™ treatment for 45 days. As expected, the levels of both FSH and LH were increased after chemotherapy whereas progesterone, estrogen and AMH levels were decreased. XAR™ treatment to chemoablated mice led to a statistical decrease (*p* < 0.0001) in FSH levels and an statistical increase (*p* < 0.001) in AMH levels. When XAR™ was given for 30 days along with chemotherapy (preventive treatment group) the effect was more significant with maximum levels of AMH (*p* < 0.001). In males, the testosterone levels decreased after chemotherapy and were near normal when XAR™ was given for 15 days after chemotherapy and improved further when XAR™ was given for 30 days along with chemotherapy (Preventive group). There was no statistical difference in testosterone levels of curative treated, preventive treated and untreated control groups suggesting attenuation and reversal of the chemoablation. Sperm parameters (sperm count, mobility and viability) reduced drastically after chemotherapy and were restored to near normal values after XAR™ treatment (in both curative treatment and preventive treatment group) (Table 1C).

### Effect of XAR™ treatment on the histology of ovaries and testes

Microscopic examination of ovarian sections revealed that ovaries from the control group exhibited normal histological structure at different stages of follicle development (Fig. 3). The number of follicles appeared much more after XAR™ treatment (B) compared to untreated control (A) in agreement with the data of follicle counts shown in Table 1A. Chemoablation led to the loss of ovarian follicles (Fig. 3C, E) and follicles in different stages of development were seen as a result of XAR**™** treatment to the chemoablated ovaries (Fig. 3D, F). Loss of follicles in chemoablated ovaries is well known in literature but it was of interest to observe a stimulatory effect of XAR™ on follicle numbers in both intact and chemoablated ovaries.

**Fig. 3:** Effect of chemoablation and XAR™ treatment on ovarian and testicular histology. **A** Untreated control (Ovary); **B** XAR™ treated (Ovary); **C** Bu-Cy Curative control (Ovary); **D** Bu-Cy-XAR™ Curative treatment (Ovary); **E** Bu-Cy Preventive control (Ovary); **F** Bu-Cy-XAR™ Preventive treatment (Ovary); **G** Untreated control (Testis); **H** XAR™ treated (Testis); **I** Bu Curative control (Testis); **J** Bu XAR™ Curative treatment (Testis); **K** Bu Preventive control (Testis); **L** Bu XAR™ Preventive treatment (Testis). In ovaries, treatment for 45 days resulted in large number of follicles in different stages of development. Follicles reduced after chemotherapy were restored after XAR™ treatment in both curative and preventive groups. In testis, normal spermatogenesis was observed in untreated control and after XAR™ treatment whereas germ cells loss was noted after chemotherapy with Bu. XAR™ treatment completely restored spermatogenesis and pre-treatment with XAR™ prevented germ cells loss

The untreated control and XAR™ treated mice testes showed normal histology consisting of well-organized seminiferous tubules exhibiting spermatogenesis and regular interstitial connective tissue. An increase in germ cells numbers per tubule was observed after XAR™ treatment (H) compared to untreated control (G). The testes had a well-organized pattern of spermatogenesis with radially arranged sperm along-with Sertoli cells and exhibiting different stages of differentiation of spermatogonial cells (Fig. 3). A loss of germ cells was noted after chemotherapy with minimal spermatogenesis (I & K). Sertoli cells collapsed due to the absence of germ cells. XAR™ treatment resulted in regeneration of testis wherein spermatogenesis was observed in all the tubules compared to chemotherapy controls in both curative (J) and preventive (L) groups.

### Differential expression of pluripotent transcripts in adult gonads after XAR™ treatment and chemotherapy

Treatment with XAR™ (25 mg/kg) for 45 days to normal adult mice, led to increased expression of the pluripotent transcripts specific for VSELs (*Oct-4A, Sox-2, Nanog) *and primordial germ cell *(Stella, Fragilis*) in both the ovaries and testes (Fig. 4). As reported earlier, we observed increased expression levels of the transcripts in chemoablated gonads (26,32). Results suggest a direct stimulatory action of XAR**™** on the gonadal stem cells.

**Fig. 4:** Effects of XAR™ and chemotherapy treatment on pluripotent transcripts in adult gonads. Differential expression of transcript levels in (**A**) ovary and (**B**) testes was seen on treatment with XAR™, Bu-Cy and Bu. Compared to control, mice treated with XAR™ showed significant increase in expression of *Oct-4A, Sox-2, Nanog, Stella, and Fragilis* transcripts, both in ovaries and testis. Two-way ANOVA was used for statistical analysis, ****p < 0.0001, ***p < 0.001, **p < 0.01, *p < 0.05

## Effect of XAR™ treatment on ovarian transcripts of interest by quantitative RT-PCR

Both pluripotent (*Oct4A, Sox2, Nanog*) and primordial germ cell (Stella, Fragilis) specific markers were found to be upregulated after XAR™ treatment to chemoablated mice in the curative group. In the preventive group, where XAR™ was administered for 2 days prior to chemotherapy, expression of these transcripts remained unaffected and rather showed a slight upregulation. Various transcripts specific for the progenitors (OSCs) (*Total Oct-4, Sca1*) and pre-meiotic germ cells (*Mvh, Stra-8*) and oocytes (*Nobox, Hoxa10*) showed increased expression after XAR™ treatment to chemoablated mice in the curative group (Fig. 5). This was accompanied by increased expression of meiotic (*Scp3, Dmc1*) and proliferation (*Pcna*) markers. In agreement with an earlier report by Patel et al. [28] we observed that alternately spliced *Fshr3* transcripts showed increased regulation whereas canonical *Fshr1* was found to be minimally affected by XAR™ treatment. XAR™ treatment also resulted in increased expression of *Sirt1, Sirt6, p53* and *Nampt* (required for maintaining the redox potential). Results show that treatment of chemoablated mice later on with XAR™ led to resumption of neo-oogenesis from the VSELs and OSCs present in the ovary in an effective manner followed by PF formation.

**Fig. 5:** Effect of chemoablation and XAR™ treatment on transcripts in ovary. XAR™ treatment in chemoablated mice led to significant increase in expression of transcripts specific to (**A**) pluripotent cell – *Oct-4A, Sox-2, Nanog*, primordial germ cell – *Stella, Fragilis*, (**B**) progenitor OSCs – *total Oct-4, Sca1*, pre-meiotic germ cells – *Mvh, Stra-8*, oocytes – *Nobox, Hoxa-10*, (**C**) *Fshr – Fshr1, Fshr3*, meiotic – *Scp3, Dmc1*, proliferation (*Pcna*), (**D**) maintaining redox potential – Sirt1, Sirt6, p53, and Nampt. The findings are suggestive of XAR™ treatment reinstating neo-oogenesis from VSELs and OSCs in ovary. One-way ANOVA was used for statistical analysis of curative control vs curative treatment and preventive control vs preventive treatment group, ****p < 0.0001, ***p < 0.001, **p < 0.01, *p < 0.05

### Effect of XAR™ treatment on testicular transcripts of interest by quantitative RT-PCR

Similar to the ovaries, XAR™ treatment to chemoablated testes also resulted in the up-regulation of both pluripotent (*Oct-4A, Sox-2, Nanog*) and primordial germ cells (*Stella, Fragilis*) specific transcripts. The fold increase was much more in the testes (10–30 folds) compared to the ovary (10–15 folds) which is expected since the rate of spermatogenesis is much more compared to oogenesis (Figs. 5A and 6A). An increase was noted in the transcripts specific for ‘progenitors’ SSCs (*total Oct-4, Sca1*) and germ cells (*Gfra, Mvh, Dazl, c-Kit*). Increased expression of markers suggestive of meiosis (*prohibitin, protamine, Scp3*) and spermatids (*Cyclin B1*) was also observed. Similar to ovaries and earlier published data on adult mouse testes [29], alternately spliced *Fshr3* was more markedly regulated by XAR™ rather than the canonical *Fshr1*. A similar pattern of increased expression of *Sirt1, Sirt6, p53* and *Nampt* was observed in the testes after XAR™ treatment (Fig. 6). Results show that treatment of XAR™ restored spermatogenesis in the chemoablated testes in an effective manner.

**Fig. 6:** Effect of chemoablation and XAR™ treatment on transcripts in testes. The expression of transcripts specific to (**A**) pluripotent cell – *Oct-4A, Sox-2, Nanog*, primordial germ cell – *Stella, Fragilis*, (**B**) progenitor SSCs – *total Oct-4, Sca1*, germ cells – *Gfra, Mvh, Dazl, c-Kit*, (**C**) *Fshr – Fshr1, Fshr3*, meiotic—prohibitin, protamine, *Scp3*, spermatids – *Cyclin B1*, proliferation (*Pcna*), (**D**) maintaining redox potential – *Sirt1, Sirt6, p53*, and *Nampt* were significantly altered on XAR™ treatment. XAR™ treatment reinstated spermatogenesis in chemoablated testes. One-way ANOVA was used for statistical analysis of curative control vs curative treatment and preventive control vs preventive treatment group, ****p < 0.0001, ***p < 0.001, **p < 0.01, *p < 0.05

### Effect of XAR™ treatment on Oct-4A/Oct-4 ratio

Two populations of stem cells exist in all adult tissues and gonads including the pluripotent VSELs and tissue committed progenitors (e.g. ovarian stem cells OSCs in the ovary and spermatogonial stem cells SSCs in testes) [30, 31]. Being pluripotent, VSELs express nuclear Oct-4A and OSCs/SSCs express cytoplasmic Oct-4. It is interesting to note that the Oct-4A/Oct-4 ratio was increased by two-fold (p < 0.001) after chemoablation in both ovary and testes (Fig. 7) indicating chemotherapy destroyed follicular reserve and sperm along with the OSCs / SSCs. However, VSELs survived chemotherapy because of their quiescent nature as reported earlier [11, 26, 32]. The results suggest that nuclear Oct-4A positive cells persisted whereas the cytoplasmic Oct-4 positive OSCs were selectively destroyed by chemotherapy. This ratio of Oct-4A/Oct-4 was restored when chemoablated gonads were treated with XAR™.

**Fig. 7:** Effect of XAR™ treatment on OCT-4A/Oct-4 ratio in gonads. The ratio of Oct-4A/Oct-4 in (**A**) ovary (**B**) and testis increased by two-fold in chemoablated gonads as compared to untreated control, whereas XAR™ treatment of chemoablated mice showed restored levels of Oct-4A/Oct-4. Two-way ANOVA was used for statistical analysis, ****p < 0.0001, ***p < 0.001, **p < 0.01, *p < 0.05

### Effect of XAR™ treatment on antioxidant indices

XAR™ treatment increased the expression of GSH and SOD and decreased MDA as shown in Fig. 8. Malondialdehyde (MDA) is an end product of lipid peroxidation, and increased MDA levels along with decreased GSH and SOD levels reflect oxidative stress [33]. In contrast, increased levels of GSH and SOD indicate tissue healing after oxidative damage [34, 35]. Oxidative stress leads to ovarian failure by inhibiting nuclear and cytoplasmic maturation of oocytes and inducing apoptosis [34]. Chemotherapy (with Cy + Bu in female and Bu in male mice) resulted in more than two-fold reduction (*p* < 0.0001) in GSH and SOD levels whereas MDA levels were increased by two-fold (*p* < 0.0001). XAR™ treatment for 15 days resulted in the recovery of GSH, SOD and MDA levels (*p* < 0.0001). Pre-treatment with XAR™ prevented chemotherapy-mediated decrease of GSH and SOD levels and also impacted MDA levels as compared to untreated control.

**Fig. 8:** Effect of chemotherapy and XAR™ treatment on antioxidant indices (**A**) GSH (**B**) MDA and (**C**) SOD in testis and ovaries. The curative and preventive groups treated with chemotherapy—Busulfan-Cyclophosphamide in female mice and Busulfan in male mice, led to decreased GSH, SOD levels and increased MDA levels. However, XAR™ treatment led to increased GSH, SOD levels and decreased MDA levels. In addition, the antioxidant indices increased in chemoablated XAR™ treated curative and preventive group, indicating increased tissue healing in oxidative damage. Two-way ANOVA was used for statistical analysis, ****p < 0.0001, ***p < 0.001, **p < 0.01, *p < 0.05

## Discussion

In the present study, we show that XAR™, similar to FSH, successfully stimulated the growth of ovarian follicles and also improved ovarian reserve including an increase in the numbers of primordial follicles. AMH levels, which mark the ovarian reserve [36, 37], were increased to a greater extent after XAR™ treatment on D7 compared to FSH treatment. Furthermore, XAR™ provided both curative and protective effects on the gonads when adult male and female mice were exposed to chemotherapy. It successfully regenerated and restored gametogenesis in chemoablated ovaries and testes and also prior treatment with XAR™ offered protection to the gonads from the adverse effects of chemotherapy. The study highlights a possible use of XAR™ for cancer patients to protect their gonads from the deleterious effects of oncotherapy and also to regenerate their non-functional gonads after exposure to various cancer drugs which are known to adversely affect fertility. Results need to be confirmed on human gonads and by others working in the field. For the sake of clarity, we have divided the discussion under various subheadings.

### Effect of XAR™ compared to FSH on ovarian follicles

It has earlier been reported that receptors for FSH are expressed on the stem cells and that FSH directly stimulates the stem cells in both the ovaries and testes to undergo proliferation followed by differentiation [28, 38]. These stem cells include the pluripotent VSELs along with tissue-specific ‘progenitors’ OSCs in the ovary and SSCs in the testes. Thus, it was logical to study whether XAR™, similar to FSH, activated ovarian stem cells. Results show that besides the numbers of growing and antral follicles, both FSH and XAR™ increased the ovarian reserve- number of primordial follicles and that XAR™ treatment led to a greater increase in the numbers of PF on D7 compared to FSH. This was mirrored by increased AMH values after XAR™ treatment compared to FSH. Treatment of normal adult female mice with XAR™ resulted in a distinct increase in VSELs specific transcripts suggesting a direct stimulation of ovarian stem cells by XAR™ treatment. Increased primordial follicles numbers is suggestive of postnatal oogenesis and PF assembly from the stem cells and that XAR™ exerts a stronger effect compared to FSH. It can be possibly used to stimulate the ovarian follicles in infertile women in IVF Clinics. It will be cost-effective and will help make IVF services more affordable in developing countries.

Recently there is a lot of stress on treating idiopathic male infertility patients with FSH [39, 40]. Such cases will also possibly benefit from treatment with XAR™. A distinct increase in numbers of germ cells was clearly evident after XAR™ treatment to adult male mice (compare Fig. 3 G & H) along with a distinct upregulation of VSELs specific pluripotent transcripts. Results are compelling enough to undertake pilot studies to evaluate the potential of XAR™ to treat infertility.

Results of the study provide evidence to support neo-oogenesis from stem cells and primordial follicles assembly in female mice. This increase in the number of PF is a paradox to the current understanding that a female is born with a fixed number of follicles and that their number decrease with age leading to menopause. Evidence to support neo-oogenesis from stem cells on regular basis across estrus cycle in adult mice ovaries under normal physiological conditions was recently published [41]. An increase in the number of PF after treatment with both XAR™ and FSH supports the assembly of newly formed follicles possibly from the stem cells. A similar increase in number of cohorts of PF was earlier reported when mice were treated with PMSG [42]. There was an increase in VSELs, germ cells and meiosis specific transcripts suggesting differentiation of VSELs into oocytes and primordial follicle assembly in the chemoablated ovary after treatment with XAR™. There was more than 15 folds increase in *Nobox* which is an oocyte-specific transcription factor and plays a critical function during early folliculogenesis [43]. *Stella* and *Fragilis* are specific markers for PGCs and expressed on the VSELs that survive chemotherapy as reported earlier [38, 44] and were also up-regulated when chemoablated ovaries were treated with XAR™. Meiosis specific transcripts were also upregulated. However, an increase in meiosis specific markers is not expected in adult ovaries if they have a fixed number of follicles at birth. Increase in *Hoxa10, NOBOX, Scp3* and *Stra8* expression suggested increased numbers of PF on treatment with XAR™ from the ovarian stem cells. Similar to the ovaries, even chemoablated testis showed activation of the stem cells (increased expression of pluripotent and PGC specific markers) and their differentiation (increased expression of germ cells and meiosis specific markers) on the treatment of chemoablated mice with XAR™. Tripathi et al. [22] earlier reported a direct stimulatory effect of XAR™ on stem cells in peripheral blood.

Currently held view is that receptors for FSH are expressed on the Granulosa cells in the ovaries and on the Sertoli cells in the testes [45]. FSH acts indirectly on the germ cells via the canonical Fshr1 via cAMP pathway. Four different alternately spliced FSHR isoforms have been reported [46]. FSHR has also been reported on the stem cells in ovary [28, 47], testis [29], uterus [48, 49] and in the hematopoietic system [50, 51]. FSH possibly acts directly on the stem cells via growth factor type I alternately spliced transcript Fshr3 via MAPK rather than the canonical Fshr1. Fshr3 was reported to be the most predominant transcript in sheep ovarian follicles rather than the canonical Fshr1 [47]. Results of the present study showed that XAR™ exerted differential upregulation of Fshr3 rather than the canonical Fshr1. It was intriguing to note that Fshr3 was distinctly regulated by XAR™ treatment rather than the canonical Fshr1. Earlier studies have reported similar results that alternately spliced Fshr3 is modulated in association with the stem cells activity in both the ovary [28] and testes [29]. These results of direct action of FSH on tissue-resident stem cells via Fshr3 rather than canonical Fshr1 were recently reviewed [23, 24].

Resveratrol is also reported to affect ovarian and testicular biology. Resveratrol has been reported to preserve the ovarian follicle pool by increasing serum anti-müllerian hormone (AMH) levels [52]. Resveratrol has been demonstrated to relieve oogonial stem cells loss along with attenuating the effect of Bu/Cy-induced oxidative apoptosis in mouse ovaries, which may be attributed to the attenuation of oxidative levels in ovaries [18]. Bezerra et al., [53] discovered that resveratrol promotes primordial follicle activation by reducing DNA fragmentation and stimulates granulosa cell proliferation [53]. Recently, Jiang et al., [54] reported that resveratrol treatment in POF model increased expression levels of *Mvh* and *Oct-4* indicating that resveratrol significantly prompted the proliferation of germline stem cells in the POF model which is similar to our finding [54]. Similarly, Resveratrol has been reported to exert beneficial effects on testes to ameliorate the loss of spermatogonial stem cells (SSCs) in busulfan-induced infertile mice [55]. Resveratrol has been reported to improve sperm motility, function and numbers along with enhancing antioxidant defences in the testes [56, 57].

A proof-of-principle trial can be undertaken using XAR™ to treat infertile men and women.

#### VSELs survive chemotherapy in the ovary and testes

Results of the present study show that VSELs survive in chemoablated, adult mouse ovaries as well as testes. More than 15 folds increase in expression of transcripts specific for pluripotent VSELs (Oct-4A, Sox-2 and Nanog) and primordial germ cells (Stella, Fragilis) was evident in chemoablated gonads. Such a high increase is because of the dramatic loss of all other cell types in the chemoablated gonads and VSELs that make up less than 1% of total cells in the normal gonads, increase in proportion due to loss of other actively dividing cells. Thus flow cytometry data will be required to show the exact change in their numbers but surely VSELs survive chemotherapy. It has been reported earlier in mice [26, 29, 32] and humans [58, 59] that VSELs survived oncotherapy in both ovary and testes. Ratajczak’s group has reported that VSELs survive total body irradiation in the mouse bone marrow [60]. VSELs are the most primitive and pluripotent stem cells that exist in multiple adult tissues and remain quiescent in nature. They undergo rare asymmetrical cell divisions to self-renew occasionally and give rise to slightly bigger progenitors including OSCs in the ovary and SSCs in the testes. Underlying mechanisms to explain their quiescent nature have also been reported [61].

In our study, chemotherapy resulted in significant exhaustion of antioxidant potential as evident by depleted GSH and SOD levels along with high MDA levels in both ovaries and testis. XAR™ treatment resulted in the recovery of GSH and SOD levels and in preventive groups an increased level of GSH and SOD resulted in the protection of the ovary and testis from the deleterious impact of chemotherapy induced damage. A similar mechanism of upregulated antioxidant mediated protection has been reported earlier [62, 63]. Li and Liu, [64] has reported that resveratrol treatment improved ovarian function in the POF model by decreasing MDA and increasing SOD levels [64]. Resveratrol has been known as a SIRT1 activator [65] and was reported to enhance progesterone secretion and luteinization-related genes expression in the ovary by stimulating the expression of SIRT1 in granulosa cells [66]. The reduction of ovarian SIRT1 mRNA expression induced by chemoablation in our study is coherent with other reported studies wherein SIRT1 expression is significantly down-regulated in premature ovarian failure [52]. Resveratrol has also been reported to preserve the entire ovarian follicle pool by increasing serum anti-müllerian hormone (AMH) levels [52]. Our findings suggest that XAR™ restores ovarian function through increasing AMH level and diminishing ovarian inflammation, predominantly via upregulation of SIRT1 expression, which is also reported by Said et al., [52].

#### Curative effects of XAR™ on adult ovary and testis

Results of the present study clearly delineate the curative potential of XAR™ on non-functional gonads of chemoablated mice. Germ cell loss was clearly evident after chemotherapy in both ovary and testis accompanied by elevated FSH levels and reduction of sex steroids. In female mice, a reduction of AMH values was observed whereas sperm count was markedly reduced after chemotherapy. XAR™ treatment (25 mg/kg b.w. for 15 days) resulted in normalization of FSH and sex steroid levels along with AMH and sperm count. XAR™ treatment resulted in the presence of follicles in chemoablated ovaries (Fig. 3D) and spermatogenesis (Fig. 3J) was apparently restored in the testes. The qRT-PCR study enabled us to track neo-oogenesis and spermatogenesis in chemoablated gonads after XAR™ treatment.

In the ovaries, there was a marked increase in both VSELs (*Oct-4A, Sox-2, Nanog*) OSCs (*total Oct-4, MVH, Stella, Fragilis*) and oocyte (*Nobox, Hoxa10*) specific markers after XAR™ treatment accompanied by an increase in proliferation (*Pcna*) and meiotic (*Scp3, Dmc1*) markers. This clearly suggested that XAR™ treatment stimulated the VSELs to increase in numbers and undergo further differentiation into oocytes followed by primordial follicle assembly. Stra-8 is a crucial pre-meiotic germ cell marker [67] whose transcripts are not expected to be expressed in adult ovaries if a female has a fixed ovarian reserve by birth. More than 5–7 folds increase in Stra-8 transcripts provide strong data in support of neo-oogenesis from stem cells in adult ovaries and this process is supported by XAR™. Neo-oogenesis does occur from the stem cells in adult ovaries and the results of the present study provide a paradigm shift in the current belief that females are born with fixed numbers of follicles by birth.

In the testes, similar to the ovaries, there was a marked increase in the expression of pluripotent transcripts specific for VSELs (*Oct-4A, Sox-2, Nanog*), SSCs (*TOct-4, Stella, Fragilis*), germ cells (*Mvh, Dazl, Gfra*), proliferation (*Pcna*), meiosis (*Scp3*, Prohibitin) and spermatids (*cyclin B1*, Protamine). Results suggest a complete restoration of spermatogenesis from the VSELs that survived chemotherapy on exposure to XAR™.

In both the ovaries and testes, XAR™ treatment increased the expression of *Sirt 1, Sirt 6* and *Nampt* and *p53* values. Sirtuins belong to a well-conserved family of NAD^+^ dependent enzymes that respond to a variety of stresses and are emerging as key anti-aging molecules and regulators in many diseases [68]. Sirtuins have been reported to prevent oxidative threat to fertility by modulating the antioxidant balance of the cell [69, 70]. Increased expression levels of SIRT1 and SIRT6 in testis and ovaries on treatment with XAR™ to chemoablated mice were also intriguing. SIRT1 and SIRT6 represent ovarian reserve as well as anti-Müllerian hormone (AMH), antral follicle counts (AFC), and follicle stimulating hormone (FSH) levels in the clinical assessment of ovarian function [71]. In humans, XAR™ treatment has been reported to increase hemopoietic stem cells, mesenchymal stem cells and endothelial progenitor cells [22].

To conclude, XAR™ treatment can regenerate chemoablated ovaries and testes by restoring the proliferation/ differentiation of endogenous stem cells resulting in gametogenesis.

#### Protective effects of XAR on adult ovary and testis

Administration of XAR™ for two days prior to chemotherapy successfully protected the gonads from the damaging effects. Circulatory levels of FSH, steroid hormones remained near normal and histological analysis of both ovaries and testes revealed normal histology with intact follicles and spermatogenesis respectively. qRT-PCR data in both the ovaries and testes revealed normal (or slightly increased) expression of stem/progenitor cells and gametogenesis specific transcripts. To conclude, XAR™ treatment can protect the gonads from the adverse effects of chemotherapy.

Well-designed clinical trials are now needed to study the preventive and curative effects of XAR™ among cancer patients/ survivors.

## Conclusions

To conclude, XAR™ exerts effects similar to FSH on adult mouse ovaries possibly by a direct action on endogenous VSELs and OSCs which undergo regular differentiation (neo-oogenesis) leading to increased numbers of primordial and other growing follicles. Similarly, numbers of germ cells were increased in testes after XAR™ treatment. XAR™ provided both protective and curative effects in response to chemotherapy in mice. New follicle assembly occurred from the stem cells on treating chemoablated mice with XAR™. The study model can be further used to study neo-oogenesis and follicle assembly in the adult ovary. The results also have translational potential and warrant well designed pilot clinical studies to evaluate if XAR™ could be used to stimulate ovaries similar to FSH. The advantage will be the costs involved, XAR™ is much cheaper compared to recombinant FSH, currently being used in ART clinics. Also, both preventive and curative effects of XAR™ need to be evaluated in cancer patients/survivors.

## Supplementary Information

**Additional file 1: Supplementary Table.** Detailsof primers used in the study.

## Data Availability

All the results are provided in details in the text.

## Abbreviations

AMH: Anti mullerian hormone
E2: Estradiol
FSH: Follicle Stimulating Hormone
GSH: Glutathione
LH: Luteinizing hormone
MDA: Malondialdehyde
OSC: Ovarian stem cells
PF: Primordial follicles
SOD: Superoxide dismutase
SSCs: Spermatogonial stem cells
VSELs: Very small embryonic-like stem cells
XAR™: Extremely active nano-formulation of resveratrol
